The article "Investigation on the Relationship between Sleep Quality and Depression and Anxiety in Hospitalized Patients with Different Levels of AECOPD" was retracted in 2023. Reasons: signs of a paper mill; unreliable results or conclusions.

# Investigation on the Relationship between Sleep Quality and Depression and Anxiety in Hospitalized Patients with Different Levels of AECOPD

**DOI:** 10.1155/2022/5901552

**Published:** 2022-04-30

**Authors:** Dingfang Liu, Ying Zou, Yumei Wang

**Affiliations:** Department of Respiratory and Critical Care Medicine, No.6th People's Hospital Affiliated to Shanghai Jiao Tong University School, Shanghai 200233, China

## Abstract

**Purpose:**

To explore the correlations between sleep quality and depression and anxiety in hospitalized patients with acute exacerbation of chronic obstructive pulmonary disease (AECOPD).

**Methods:**

A total of 131 AECOPD patients treated at No.6th People's Hospital affiliated to Shanghai Jiao Tong University School from January 2018 to December 2020 were selected and divided into the classes I (*n* = 30), II (*n* = 23), III (*n* = 37), and IV (*n* = 41) based on the severity of AECOPD. The Pittsburgh sleep quality index (PSQI) and the hospital anxiety and depression scale (HADS) were employed to assess the quality of sleep and anxiety/depression in AECOPD patients. The Pearson correlation analysis explored the associations between PSQI score and HADS anxiety/depression score. Binary logistic regression was utilized to determine risk factors for anxiety/depression in AECOPD patients.

**Results:**

The PSQI score, HADS anxiety score, and HADS depression score in patients with AECOPD class III and class IV were significantly higher than those of classes I and II. The severe anxiety and depression ratio were significantly different among patients with classes I–IV AECOPD. The severity of AECOPD was significantly correlated with the PSQI score (*r* = 0.51, *P* < 0.001), HADS anxiety score (*r* = 0.66, *P* < 0.001), and HADS anxiety score (*r* = 0.65, *P* < 0.001). Binary logistic regression analysis showed that the COPD duration, the severity of AECOPD, and PSQI score were the risk factors for anxiety and depression in patients with AECOPD.

**Conclusions:**

Poor sleep quality, anxiety, and depression are common in patients with AECOPD. Improvement of sleep quality may help to alleviate anxiety and depression in AECOPD patients.

## 1. Introduction

Chronic obstructive pulmonary disease (COPD) is a chronic respiratory disease characterized by reversible airflow restriction. The prolonged course of the disease often leads to the decline of activity tolerance, the loss of independence, and the decline of social function, which seriously affects patients' health and life treatment [1]. In addition, acute exacerbation of chronic obstructive pulmonary disease (AECOPD) is a common reason for COPD patients, which causes a severe burden on patients and their families. Studies [2, 3] found that sleep disorders are common in patients with AECOPD, such as shortened sleep time, disordered sleep structure, and increased midway wake-up. However, the prevalence of sleep disorders in patients with different levels of AECOPD is not apparent. At present, the specific mechanism of sleep disorder in patients with AECOPD is still unclear. A study [4] speculates that it is related to nocturnal airflow obstruction, reduction of arterial oxygen saturation, hypercapnia, and auxiliary respiratory muscle fatigue caused by the disease itself. Other indicated that it may also be related to emotional disorders and adverse effects emotions such as anxiety and depression. Research [5] founds that anxiety and depression in AECOPD patients can be superimposed on sleep disorders, which can synergistically affect the overall health level of patients. In addition, sleep disturbance has been confirmed to be one of the inducements of AECOPD that can be improved [6], and improving the quality of life of AECOPD patients by improving sleep status has broad clinical application prospects. This study intends to explore the status of sleep quality, anxiety, and depression in patients with AECOPD at different levels and clarify the relationship between them, which will help to establish the diagnosis and treatment system of physical and mental status and quality of life of hospitalized AECOPD patients and strengthen the overall management level of AECOPD complications in the clinic.

## 2. Methods

### 2.1. Research Objects

This study prospectively enrolled 131 hospitalized patients with AECOPD in our department from January 2018 to December 2020. The inclusion criteria were precise diagnosis of AECOPD and compliance with the 2017 China guidelines for chronic obstructive pulmonary disease, patients with dyspnea, cough, and expectoration exceeding daily variation, and excluding pulmonary infection, congestive heart failure, pleural effusion, pneumothorax, etc. disease. Exclusion criteria are as follows: (1) In addition to AECOPD, the patients also have other major diseases, such as malignant tumors, severe liver and kidney insufficiency, chronic heart failure, and end-stage renal disease; (2) the patient had schizophrenia and other mental disorders in the past or was taking antipsychotics within 3 months before enrollment; and (3) the patient refused to participate in the study. The study was approved by the Ethics Committee of No.6th People's Hospital affiliated to Shanghai Jiao Tong University School [No.: 2018-KY-017(K)], and informed consent was provided by all participants.

### 2.2. Research Methods

According to the criteria of China's guidelines for chronic obstructive pulmonary disease in 2017, AECOPD patients are divided into classes I, II, III and IV. Of these classes, I is the lightest, and grade IV is the heaviest. Two specialist nurses conducted a questionnaire survey on the patients, including the patient's age, gender, course of COPD, education level, marital status, payment method of medical expenses, severe cough at night, and hemoptysis.

Pittsburgh Sleep Quality Index (PSQI) was used to evaluate the sleep quality of hospitalized patients with AECOPD [7]. In 1996, Liu Xianchen, a domestic scholar, tested the reliability and validity of the Chinese version of the scale and considered it suitable for domestic patients. It is one of the most widely used investigation and research scales for sleep quality evaluation and curative effect observation for patients with sleep disorders and mental disorders. The total score on the scale is 21. The higher the score, the worse the sleep quality.

Patients' anxiety and depression status were evaluated by the General Hospital Anxiety and Depression Scale (HADS) [8]. The scale is mainly used to screen anxiety and depression in general hospital patients. Domestic scholars, Sun Zhenxiao and others, tested the reliability and validity of its Chinese version, suggesting that the results are good in domestic inpatients. The HADS scale is divided into two subscales: anxiety and depression. Each scale has 7 items, with a score of 0-3 for each item and a total score of 21 points. It is generally believed that anxiety or depression exists when the score is ≥8.

### 2.3. Statistical Analysis

SPSS 22.0 Chinese version software was used for statistical analysis. The measurement data of normal distribution were expressed as mean ± standard deviation, and one-way ANOVA and Tukey posttest carried out the multi-group comparison and pairwise comparison. The counting data were expressed in frequency and percentage, and the chi-square test compared the groups. The correlation coefficient between the two variables was determined by Pearson correlation. Binary logistic regression was used to determine the risk factors of anxiety and depression. Bilateral test *α* = 0.05.

## 3. Results

### 3.1. General Characteristics of Patients

A total of 131 patients were included in this study, of which 30 (22.90%), 23 (17.56%), 37 (28.24%), and 41 (31.30%) were classes I, II, III, and IV patients, respectively. The course of class III and IV COPD was significantly longer than class I patients. There was no significant difference in age, gender composition, education level, marital status, payment method of medical expenses, nighttime cough, and hemoptysis among classes I-IV patients (all *P* > 0.05) (see Table 1).

### 3.2. PSQI and HADS Scores of Patients with AECOPD at Different Levels

The PSQI score, HADS anxiety score, and HADS depression score of classes III and IV AECOPD patients were significantly higher than those of classes I and II patients. The proportion of classes I-IV anxiety was 16.67%, 60.87%, 81.08%, and 85.37%, while the ratio of depression was 16.67%, 56.52%, 67.57%, and 63.41%, respectively. There was a significant difference in the proportion of patients with severe anxiety and depression in classes I-IV (see Table 2).

### 3.3. Correlation between Disease Class of AECOPD Patients and PSQI and HADS Scores

The correlation analysis indicated that the severity class of COPD was significantly correlated with PSQI score (*r* = 0.51, *P* < 0.001), HADS anxiety score (*r* = 0.66, *P* < 0.001), and HADS depression score (*r* = 0.65, *P* < 0.001) (see Table 3 and Figure 1).

### 3.4. Univariate and Multivariate Analysis

Taking whether the patient has anxiety/depression as the dependent variable, the binary logistic regression showed that the course of COPD and the grading of AECOPD were the risk factors of anxiety and depression (see Table 4).

## 4. Discussion

COPD is a prevalent chronic respiratory disease in elderly patients. It has the characteristics of high incidence rate, long duration of illness, and heavy family burden. COPD can cause clinical symptoms such as cough, expectoration, and asthma and have a significant impact on the mental health of patients [9]. However, there were few reports on the relationship between clinical severity and patients' mental health. In this study, we investigated the effects of AECOPD on anxiety, depression, and sleep quality.

Through the HADS scale, we found that anxiety and depression were more common in the AECOPD population, and the prevalence increased with the aggravation of the disease. Literature [10] reported that anxiety and depression often coexist in patients with COPD. In fact, the prevalence of anxiety and depression in patients with stable COPD is 10%-24% and 10%-19%, respectively [11, 12], which is lower than the level reported in this study. This study mainly focuses on AECOPD patients, whose condition is often dangerous and even life-threatening. This acute stress response may increase the anxiety and depression of patients. In addition, anxiety and depression are also risk factors for repeated hospital admissions in the short-term in patients with AECOPD, which seriously increases the pressure and medical burden of patients and forms a vicious circle [13].

PSQI scale results show that the decrease of sleep quality is also a common phenomenon in AECOPD patients, which may be related to cough and expectoration at night, hypoxemia, and paralysis of the respiratory regulation center [14]. Akinci et al. [15] found that more than 94% of patients with moderate and severe COPD had a PSQI >5, which is similar to the results of this study. Another study has found that poor sleep quality is an independent risk factor for the acute attack of COPD [16]. Therefore, paying attention to patients' sleep quality may help improve the condition of COPD.

This study first reported that poor sleep quality in patients with AECOPD is a risk factor for anxiety and depression, not reported in the previous literature. In patients with stable COPD, a study has found that the HADS anxiety and depression scores of patients with poor sleep quality are significantly higher than those with good sleep quality [17]. In addition, this study also found that the course and severity of COPD were related to anxiety and depression. Koulouris et.al found that COPD duration and pulmonary function were independent risk factors affecting patients' psychological disorders [18].

Based on the results, we speculate that the following medical and nursing measures may help improve the anxiety and depression of AECOPD patients: First, actively improve the condition through oxygen inhalation, resolving phlegm, antispasmodic, auxiliary ventilation, and other treatments. Some studies [19, 20] pointed out that admission to the intensive care unit can significantly increase patients' anxiety and depression, while transfer to the general ward can help alleviate patients' emotions. Secondly, improving the sleep quality of AECOPD patients through the rational use of sedatives, antitussive, and other active treatments may help to reduce anxiety and depression. Economou et.al [21] investigated the anxiety and depression of COPD patients before and after treatment and found that the anxiety and depression of patients can be continuously improved after improving sleep quality. Finally, through multi-team cooperation, enhancing patients' confidence in overcoming diseases may help to improve patients' mood.

In conclusion, this study explored the relationship between the severity of disease, sleep quality, anxiety, and depression in patients with AECOPD. It was found that the severity of disease and sleep quality were the risk factors affecting anxiety and depression. Therefore, actively treating primary diseases and improving patients' sleep quality can help to improve patients' destructive emotions such as anxiety and depression. In view of the fact that this study is a single-center study, the conclusions obtained need to be confirmed and promoted by multicenter studies.

## Figures and Tables

**Figure 1:** Correlation between the severity of AECOPD and patients' PSQI (a) and HADS score (b, c).

**Table 1:** Comparison of general characteristics of inpatients with different levels of AECOPD.

Index	I (*n* = 30)	II (*n* = 23)	III (*n* = 37)	IV (*n* = 41)	F/*χ*^2^	*P*
Age (years)	77.47 ± 8.59	74.35 ± 8.77	72.92 ± 10.07	74.80 ± 9.32	1.35	0.26
Gender (male) (case, %)	27 (90.00)	20 (86.96)	33 (89.19)	37 (90.24)	0.19	0.98
Course of COPD (years)	13.93 ± 3.00	15.22 ± 4.02	17.22 ± 5.01^a^	16.98 ± 5.29^a^	3.78	0.01
Education level					4.23	0.65
Primary school (case, %)	11 (36.67)	10 (43.48)	13 (35.14)	22 (53.66)		
Junior high school to senior high school (case, %)	14 (46.67)	10 (43.48)	18 (48.65)	12 (29.27)		
Bachelor's degree or above (case, %)	5 (16.66)	3 (13.04)	6 (16.22)	7 (17.07)		
Marital status					4.64	0.59
Unmarried (case, %)	0 (0.00)	1 (4.35)	1 (2.70)	2 (4.88)		
Divorced or widowed (case, %)	9 (30.00)	5 (21.74)	8 (21.62)	5 (12.20)		
Married (case, %)	21 (70.00)	17 (73.91)	28 (75.68)	34 (82.93)		
Payment method of medical expenses					2.37	0.50
Medical insurance (case, %)	29 (96.67)	21 (91.30)	36 (87.30)	37 (90.24)		
Self-expense (example, %)	1 (3.33)	2 (8.70)	1 (2.70)	4 (9.76)		
Nocturnal cough (case, %)	8 (26.67)	5 (21.74)	8 (21.62)	11 (26.83)	0.46	0.93
Hemoptysis (case, %)	4 (13.33)	3 (13.04)	5 (13.51)	4 (9.76)	0.34	0.95

^a^Compared with class I group, *P* < 0.05.

**Table 2:** Comparison of PSQI score and HADS anxiety/depression score in patients with different levels of COPD.

Index	I (*n* = 30)	II (*n* = 23)	III (*n* = 37)	IV (n =41)	F/*χ*^2^	*P*
PSQI (score)	8.03 ± 2.04	9.52 ± 3.12	13.08 ± 2.96^ab^	13.17 ± 4.89^ab^	17.22	<0.001
HADS anxiety (score)	5.50 ± 2.40	8.39 ± 2.74^a^	11.05 ± 3.84^ab^	13.76 ± 4.59^abc^	31.87	<0.001
No anxiety (case, %)	25 (83.33)	9 (39.13)	7 (18.92)	6 (14.63)	74.74	<0.001
Mild anxiety (case, %)	4 (13.33)	9 (39.13)	9 (24.32)	4 (9.76)		
Moderate anxiety (case, %)	1 (3.34)	5 (21.74)	16 (43.24)	11 (26.83)		
Severe anxiety (case, %)	0 (0.00)	0 (0.00)	5 (13.51)	20 (48.78)		
HADS depression (score)	4.40 ± 2.69	6.96 ± 3.94	9.86 ± 4.11^ab^	13.41 ± 4.71^abc^	32.10	<0.001
No depression (cases, %)	25 (83.33)	10 (43.48)	12 (32.43)	15 (36.59)	48.41	<0.001
Mild depression (case, %)	5 (16.67)	9 (39.13)	9 (24.32)	6 (14.64)		
Moderate depression (case, %)	0 (0.00)	3 (13.04)	11 (29.73)	11 (26.83)		
Severe depression (case, %)	0 (0.00)	1 (4.35)	5 (13.51)	19 (46.34)		

^a^Compared with class I group, *P* < 0.05. ^b^Compared with class II group, *P* < 0.05. ^c^Compared with class III, *P* < 0.05.

**Table 3:** Correlation between AECOPD severity and PSQI and HADS scores.

	PSQI score	HADS score	HADS score
AECOPD severity	0.51∗∗∗	0.66∗∗∗	0.65∗∗∗

∗∗∗*P* < 0.001.

**Table 4:** Results of multivariate binary logistic regression analysis affecting anxiety and depression in hospitalized patients with AECOPD.

Index	HADS anxiety		HADS depression		HADS anxiety		HADS depression	
	Univariate Exp (B) (95% CI)	*P* value	Univariate Exp (B) (95% CI)	*P* value	Multivariate Exp (B) (95% CI)	*P* value	Multivariate Exp (B) (95% CI)	*P* value
Course of COPD	2.53 (1.43, 4.54)	<0.001	1.22 (1.11, 1.76)	<0.001	1.96 (1.86, 2.07)	0.02	1.59 (1.32, 2.11)	0.007
COPD severity	3.11 (1.98, 6.09)	<0.001	2.87 (1.68, 4.99)	<0.001	3.40 (2.00, 5.78)	<0.001	2.89 (1.78, 4.71)	<0.001
PSQI score	4.87 (2.43, 9.43)	<0.001	3.99 (2.01, 5.55)	<0.001	4.12 (2.32, 6.44)	<0.001	3.54 (2.43, 5.43)	<0.001

## Data Availability

The data used to support the findings of this study are included within the article.
